RETRACTED

# MicroRNA-493 Suppresses Tumor Growth, Invasion and Metastasis of Lung Cancer by Regulating E2F1

**DOI:** 10.1371/journal.pone.0102602

**Published:** 2014-08-08

**Authors:** Yixue Gu, Ye Cheng, Ying Song, Zhijie Zhang, Min Deng, Chengkun Wang, Guopei Zheng, Zhimin He

**Affiliations:** 1 Cancer Research Institute and Cancer Hospital, Guangzhou Medical University, Guangzhou, Guangdong, PR China; 2 Medical School, University of South China, Hengyang, Hunan, PR China; Jawaharlal Nehru University, India

## Abstract

miRNAs have been proposed to be key regulators of progression and metastasis in cancer. However, an understanding of their roles and molecular mechanisms is needed to provide deeper insights for better therapeutic opportunities. In this study we investigated the role and mechanism of miR-493 in the development and progression of nonsmall-cell lung cancer (NSCLC). Our data indicated that the expression of miR-493 was markedly reduced in pulmonary carcinoma. The ectopic expression of miR-493 impaired cell growth and invasion in vitro and in vivo. Mechanically, miR-493 commonly directly targeted E2F1, which resulted in a robust reduction of the expression of mRNA and protein. This effect, in turn, decreased the growth, invasion and metastasis of lung cancer cells. Our findings highlight the importance of miR-493 dysfunction in promoting tumor progression, and implicate miR-493 as a potential therapeutic target in lung cancer.

## Introduction

Lung cancer is the most prevalent histological cancer subtype worldwide [1]. Because the majority of patients present with invasive, metastatic disease [2], understanding the basis of lung cancer progression is vital. Many factors, including tumor suppressors and oncogenes, are involved in pulmonary tumorigenesis or progression. [3], [4]. Recently, the classical members of protein-encoding genes have been expanded to include a type of non-protein-coding RNA molecule known as microRNA (miRNA) [5], [6], [7]. miRNAs are 19–24 nucleotides in length, and they regulate gene expression via imperfect base-pairing with complementary sequences located mainly, but not exclusively, in the 3′ untranslated regions (UTRs) of target mRNAs. Hence, miRNAs represent one of the major regulatory families of genes in eukaryotic cells, and they work by inducing translational repression and transcript degradation [8], [9]. Rapidly emerging evidence strongly suggests that miRNAs play crucial roles in tumorigenesis and progression [10], [11], [12]. For example, miR-34 reportedly prevents cancer initiation and progression in lung adenocarcinoma [13]. miRNA-218, a new regulator of HMGB1, reportedly suppresses cell migration and invasion in non-small cell lung cancer [14]. Nevertheless, further knowledge of the molecular mechanisms of miRNA is needed to provide deeper insights to develop better therapeutic opportunities for patients with lung cancer.

RETRACTED

In our recent study (Chen, et, al. unpublished paper), we used a miRNA microarray to find that miR-493 expression was markedly reduced in 95D cells, a highly metastatic lung cancer cell line, compared with HBE, an immortalized human bronchial epithelial cell line. Thus, we hypothesized that miR-493 might play an important role in lung cancer tumorigenesis and progression.

To test this hypothesis, we examined the expression of miR-493 using qRT-PCR in 6 lung cancer cell lines and 65 lung cancer tissue specimens in the present study. The data showed that the expression of miR-493 was markedly reduced in lung cancer cells and tissues. Functional in vitro and in vivo assays indicated that miR-493 inhibited lung cancer cell proliferation, invasion and metastasis by directly targeting the 3′-UTR of E2F1 to elicit a specific and robust knockdown of the protein. Our findings highlight the importance of miR-493 dysfunction in promoting tumor progression and tumorigenesis; and implicate miR-493 as a potential therapeutic target in lung cancer.

## Results

### miR-493 is downregulated in lung cancer and negatively associated with survival

To identify the dysregulation of miRNA-493 in lung cancer, we examined the expression of miR-493 using real-time PCR in 6 cell lines derived from lung cancer and one lung fibroblast line (MRC5); as well as an immortalized human bronchial epithelial cell (HBE). The data indicated that miR-493 expression was significantly reduced in lung cancer cells, especially in 95D, a highly metastatic lung cancer cell line (figure 1A). Furthermore, we compared the miRNA-493 expression levels in 65 fresh lung cancer tissues by real-time PCR. Similarly, the expression of miR-493 was significantly lower in lung cancer tissues than in corresponding normal lung tissues (figure 1B). To determine whether the downregulation of miR-493 impacts the lung cancer phenotypes or clinical pathological features, we employed a correlation analysis and found that miR-493 expression level was inversely correlated with tumor metastasis (p = 0.038), but not other pathological parameters such as the clinical stage (table 1). In addition, a Kaplan–Meier survival analysis was conducted using patient overall survival (OS, figure 1C) and disease-free survival (DFS; figure 1D) to analyze the significance of miR-493 further in terms of clinical prognosis. The results showed that patients with low miR-493 expression had a shorter mean OS and DFS than patients with high miR-493 expression (P = 0.006 for OS, P = 0.000 for DFS; figure 1C and D). These data suggest that the downregulation of miR-493 contributes to lung cancer carcinogenesis and prognosis.

RETRACTED

**Figure 1:** miR-493 expression levels are frequently downregulated in human lung cancer and associated with Prognosis. (A) The relative expression levels of miR-493 in 6 cell lines derived from lung cancer and one lung fibroblast line (MRC5), as well as an immortalized human bronchial epithelial cell (HBE) were determined by qRT-PCR. The data are presented as means ± SEM from at least 3 separate experiments.* p<0.05, **p<0.01. (B) The miR-493 expression levels in 65 paired human NSLCC and corresponding normal tissues were examined by real-time PCR, using GAPDH as an internal control. The expression value (ΔCt(N)- ΔCt(T)) represents the difference of in the miR-493 levels between normal tissue and tumor. A expression value >1 indicates that the miR-493 levels is increased in tumors. A expression value <1 indicates that the miR-493 levels is decreased in tumors. A paired t test (univariate) was used to compare the difference of between the normal group and cancer group. (C) Low levels of miR-493 correlates with shorter survival. The OS and DFS curves for all studied patients with high or lowmiR-493 expression.

**Table 1:** Analysis of the correlation between expression of miR-493 in primary NSCLC and its clinicopathological parameters.

Variable	Number of cases	expression of miR-493			P-value
		High expression	Median expression	Low* expression	
Total patients	65	15	7	43	
Age (years)					0.365
≥60	39	8	4	27	
<60	26	7	3	16	
Sex					0.450
Male	45	9	5	31	
Female	20	6	2	12	
Stage (NSCLC)					0.215
I, II	38	12	5	21	
III+ IV	27	3	2	22	
Smoking history					0.101
Never	18	7	3	8	
Ever	47				
Former	29	5	3	21	
Current	18	3	1	14	
Histology					0.511
SCC	25	7	3	15	
Adenocarcinoma	28	5	3	20	
Others	12	3	1	8	
Metastasis status					0.038
Metastasis	28	3	2	23	
No metastasis	37	12	5	20	

*Figure 1B expression value (ΔCt(N)- ΔCt(T)) >1 indicates that miR-493 levels is high in tumors. Expression value <−1 indicates that miR-493 levels is low in tumors. Expression value <1 and >−1 is median level. NSCLC: nonsmall-cell lung cancer;SCC: squamous cell carcinoma; T: tumor tissue; N: normal tissue.

### Overexpression of miR-493 impairs cell proliferation and invasion

To assess the biological effects of overexpressing miR-493 in lung cancer cells, stable ectopic overexpression cell subsets 95D/miR-493 and H1975/miR-493 and their paired control cells were constructed. A qRT-PCR analysis showed that the transfection were successful (figure 2A). We determined that the overexpression of miR-493 in 95D and H1975 cells markedly impaired cell proliferation compared with the controls using a cell growth rate assay (figure 2B), the cell cycle distribution (figure 2C) and a colony formation assay (figure 2D). In addition, we tested whether miR-493 could play a role in tumor growth using nude mice xenograft models (six mice per group). 95D cells transfected either with miR-493 or a scrambled control were transplanted into nude mice and developed into solid tumors in 25 days. However, the tumor growth was significantly reduced when miR-493 was stably expressed in 95D cells (figure 2 E). These results implied that miR-493 can strongly suppress tumor cell growth.

RETRACTED

**Figure 2:** Ectopic expression of miR-493 in lung cancer cells inhibits proliferation. A, stable ectopic overexpression of miR-493 was generated in cell subsets 95D/miR-493 and H1975/miR-493. qRT-PCR was used to verify the transfection. ** means P<0.001 (t-test). B, growth curves demonstrated that the lung cells were capable of proliferation. Cells were seeded in 12-well plates at the desired cell concentrations and maintained in medium containing 10% FBS. The absorption value of cells was measured at the indicated time points in triplicate and their growth rates were recorded. * means P<0.05 (t-test). C, The cells cycle's distribution of lung cancer cells was analyzed with a FACScan flow cytometer. The proliferation index (PI) was used to describe the potentiality of cell proliferation. PI = G2+S fraction)/(G1+G2+S)×100%. Left, the representative image of cell cycle percentage changing. Right, the statistical analysis of cell cycle percentage, data are presented as mean± SEM of 3 independent experiments * means P<0.05 (t-test). D, colony formation assays were used to determine the effect of miR-493 on long-term cell survival. Left, the area covered on each plate by the colonies was measured using an imaging system and represented as the percentage of the total area of the plate. Right, the effect of miR-493 overexpression on colony formation of lung cancer cells: each column represents a mean value of triplicate experiments in each group. Data are mean ± SEM. * means P<0.05 (t-test). E, miR-493 inhibited pulmonary tumor growth in mouse xenograft models (12 animals). Left, representative tumors isolated from mice 25 days after the subcutaneous injection of 95D cells that were stably transfected with the miR-493-expressing or control vector. Right, Data are mean ± SEM. * p<0.05, (t test).

In addition to cell growth inhibition, the effect of miR-493 on tumor invasion and metastasis was also addressed in this study. A wound-healing assay showed that miR-493 could dramatically suppress tumor cell mobility in 95D cells compared with the empty vector-transfected cells (figure 3A). Furthermore, an invasion assay was also performed. The result demonstrated that miR-493 could suppress the invasive ability of lung cancer cells (figure 3B). An experimental animal model was utilized to further investigate the suppressive effect of miR-493 on tumor metastasis, 95D/miR-493 cells were injected into the tail veins of nude mice (five mice per group). Empty vector-transfected (95D/control) cells were used as controls. The mice were killed and the lungs were excised, and the metastatic lesions of the lung were then detected using a Bruker Small Animal Imaging System (Germany) after 28 days. The fields of metastatic lesions formation in the lung were significantly reduced compared to the control group (figure 3C). Although visible metastatic nodules were not observed on the surface of the lung, metastatic lesions were detected in the lung by haematoxylin and eosin staining (figure 4D). These results indicated that miR-493 could effectively suppress tumor metastasis in vitro and in vivo.

RETRACTED

**Figure 3:** Expression of miR-493 inhibits the migration and invasion of lung cancer cells. A, scratch wound assays were conducted on 95D cells transfected with miR-493 and its paired control. The results from 3 separate assays were averaged together and graphed. *, P<0.05 (left). Representative images of the assays are shown. Original magnification: ×200 (right). B, the invasive properties of the H1975 and 95D cells were analyzed with a Transwell assay using a Matrigel-coated chamber. Migrated cells were plotted as the average number of cells per field of view from 3 different experiments, as described in the Materials and Methods. *P<0.01 (left). Representative images of the assays are shown. Original magnification: ×200 (right). C, in vivo metastasis assays were used to examine the lung metastatic ability of 95D/miR-493 cells labeled with green fluorescent protein(GFP) and its paired control cell 95D/control. Lung cancer cells were injected into the tail veins of five week- old mice. On day-28, all animals were sacrificed and the lungs were excised. The lung metastasis images were obtained with a Bruker Small Animal Imaging System. The lung tissue was then removed, fixed, paraffin-embedded, serially sectioned, and subjected to hematoxylin and eosin (H&E) staining. Left, Representation of the detected GFP signal in each of the five animals (the images were overlaid with green fluorescence and white light). Right, The metastatic field and fluorescence intensity significantly differed between the 95D/miR-493 group and the control group. D, Histological examination of pulmonary metastases from 95D/miR-493 and 95D/control cells by haematoxylin and eosin staining.

RETRACTED

**Figure 4:** E2F1 is a direct target of miR-493. A, Sequence alignment of microRNAs of the miR-493 and the E2F1 3′-UTR. The E2F1 3′-UTR contains one predicted miR-493-binding site. The seed regions of miR-493 and the seed-recognizing sites in the E2F1 3′-UTR are indicated in red. B and C, Luciferase assay of 95D cells (left-hand side) and H1975 cells (right-hand side), which were co-transfected with miR-493 and a luciferase reporter containing full length E2F1 3′-UTR (Luc-wt) or a mutant (Luc-mut) in which the nucleotides of the miR-493-binding site were mutated. An empty luciferase reporter construct was used as a negative control (Luc-ctrl). The luciferase activities were measured 48 hours post transfection. miR-493 markedly suppressed the luciferase activity in Luc-wt reporter constructs. The data are the means ±s.e.m. for separate transfections (n = 4). *P<0.05 versus scramble. D and E, miR-493 stable transfection reduces the E2F1 protein and mRNA levels. F and G, The level of miR-493 inversely correlated with E2F1 expression. F, The E2F1 expression levels were measured by immunohistochemistry in tumor tissues. These paraffin-embedded tissues specimens were the same source of 65fresh lung cancer tissue aforementioned in figure 1. A representative image of the expression levels of E2F1 in human lung tumor tissues (200×) is shown. G, data are means± s.e.m. * means P<0.05.

### miR-493 directly targets and inhibits E2F1

Based on the observation that miR-493 affects cell proliferation, invasion and metastasis, we searched for target genes of miR-493 related to motility and migration using two target scan algorithm (TargetScan and microRNA.org). A large number of different target genes were predicted. Among these candidate target genes, E2F1 was selected for further experimental validation, not only because it was identified as target of miR-493 by both databases (figure 4A), but also due to its frequent deregulation in tumor tissues [15], [16], [17]. A dual-luciferase reporter analysis showed that the co-expression of miR-493 significantly inhibited the activity of firefly luciferase that carried wild type but not mutant 3′-UTR of E2F1 (figure 4B, C) in 95D and H1975 cells, indicating that miR-493 may suppress gene expression via its binding sequence at 3′-UTR of E2F1. Moreover, the introduction of miR-493 diminished the expression of cellular E2F1 mRNA and protein (figure 4D, E). However, when inhibiting oligonucleotides against miR-493 were transfected into lung cancer cells 95D or H1975, an inverse expression pattern was not observed between miR-493 and E2F1 protein (data not shown). We presumed that this miRNA treatment contributed to the minimal endogenic expression in both lung cancer cells. Furthermore, the phenomenon was further validated by an inverse correlation between the level of E2F1 protein, indicated by immunohistochemistry staining, and the level of miR-493 expression assessed by q-PCR in the fresh lung cancer tissues used in the above analyses (figure 4F, G and figure 1B).

RETRACTED

### E2F1 contributes to the effect of suppress proliferation and invasion induced by miR-493

In addition, we constructed siRNA fragments targeting E2F1 to knock down the expression of E2F1 to investigate the contribution of E2F1 to the effect of miR-493 on these phenotypes. We found that the knockdown E2F1 could partly simulation the cell growth (figure 5 B) and cell invasion (figure 5C and D) phenotype induced by the overexpression of miR-493. Subsequently, rescue experiments were performed by overexpressing the E2F1-Δ3′- UTR vector (without an endogenous 3′- UTR) in cell expressing miR-493. The miR-493 induced downregulation of E2F1 was rescued upon the introduction of E2F1. Moreover, the overexpression of E2F1 attenuated the inhibition of cell growth (figure 5A) and invasion (figure 5C and E) caused by miR-493. These observations suggest that miR-493 specifically targets E2F1 specificity to contribute to the effect of on cell growth and invasion.

**Figure 5:** miR-493 inhibits the proliferation and invasion of lung cancer cells by targeting E2F1. A, The knock-down of E2F1 partly simulated the suppression lung cancer cells growth induced by the overexpression of miR-493 in 95D and H1975 cells. The growth curves demonstrated the capability of lung cells proliferation. The absorption value of cells was measured at the indicated time points in triplicate and their growth rates were recorded. B, Overexpression of exogenous E2F1 (without 3′-UTR of E2F1) rescued upon the proliferation suppression induced by miR-493 in 95D and H1975 cells. C, T The invasive properties of H1975 and 95D cells which were either knock-down or overexpression of E2F1were analyzed with a transwell assay using a Matrigel-coated chamber. The migrated cells were plotted as the average number of cells per field of view from 3 different experiments, as described in the Materials and Methods. The data are the mean ± SD.* means p<0.05. D and E, Representative images of the assays are shown. Original magnification: ×200.

### E2F1 regulations ERK and PI3K-AKT pathway in 95D and H1975 cells

E2F1 plays a critical role in cell-cycle progression, which in turn promotes cells proliferation and metastasis. However, the precise mechanism of E2F1 function is complex and depends on cellular context [18]. A recent study indicated that E2F1-dependent tumor progression was triggered by the activation of the cytoplasmic Ras/Raf signaling cascades, such as the PI3K-AKT [16] and MEK-ERK pathways [19], most of which regulate cell proliferation, survival and invasion [20], [21]. Thus, we investigated t whether miR-493 regulates these pathways by targeting E2F1. The upregulation of miR-493, via the transfection of miR-493, in 95D and H1975 cells decreased the phosphorylation levels of AKT and its downstream target GSK3β (figure 6A). Similarly, miR-493 also suppressed the levels of phosphorylated ERK (figure 6A). We also observed that the knockdown of miR-493 via transfection with anti-miR-493 in HBE, A549 and H1299 cells, in which the relative expression level of miR-493 was higher, increased the levels of phosphorylated AKT, GSK3b and ERK (figure 6B). These western blotting results demonstrated that miR-493 is negative regulator of the AKT and ERK pathways. Subsequently, rescue experiments were performed by overexpressing the E2F1-Δ3′- UTR vector (without an endogenous 3′-UTR) in miR-493-treated cells. The miR-493-induced downregulation of E2F1 was rescued upon the introduction of E2F1 (figure 6C), and the phosphorylation levels of AKT and ERK were altered in a similar manner. These observations suggest that miR-493 inhibits the AKT and ERK pathways by targeting E2F1.

RETRACTED

**Figure 6:** miR-493 inhibits the AKT and ERK pathways by targeting E2F1. (A) miR-493 overexpression reduced the activity of the AKT and ERK pathways in 95D and H1975 cells. (B) The knockdown of miR-493 by with anti-miR- 493 increased the activity of AKT and ERK signaling in HBE, A549 and H1299 cells. (C) miR-493 (or scramble control) transfection followed by E2F1 (or mock vector) transfection 24 hours later in 95D cells affects AKT and ERK signaling. The AKT pathway activity was measured by examining the expression of phosphorylated AKT (pAKT), whereas the EKR pathway activity was measured by examining expression of phosphorylated ERK (pERK).

## Discussion

Although a handful of studies have identified specific miRNAs involved in human tumorigenesis and progression [10], [11], [12]. We also believe more effort should be made to identify relevant miRNAs as well as the specific mechanisms by which they accomplish their specific functions, particularly with regard to the oncogenesis and progression of different types of tumors. Here, we identified that miR-493, a potentially candidate tumor suppressor miRNA [22], [23], was markedly reduced in lung cancer and that lower miR-493 expression was associated with tumor metastasis and poor prognosis (figure 1C, D and Table 1). Ectopic expression of miR-493 markedly attenuated the ability of the cells to proliferate and invade in lung cancer cells 95D and H1975 in vitro and in vivo.

RETRACTED

To date, the characterization of miR-493 function has not been extensive, although several targets have been identified with a key role in cell migration and metastasis pathways, including FZD4, Rhoc, MKK7 and IGF1R [22], [23], [24]. Here,we have identified a novel target of miR-493, E2F1. E2F1 is an important transcription factor that plays a critical role in cell-cycle progression and is tightly regulated by the retinoblastoma protein (Rb) [25]. The inactivation of Rb liberates E2F1 from the suppressive complex, which, in turn, induces the continuous expression of target genes whose products promote cell cycle progression [26]. The ectopic expression of E2F1 results in the neoplastic transformation of rodent cells [27], [28], and findings from transgenic models indicate that increased E2F1 activity is associated with tumor development in several tissues [29], [30], [31]. Abnormalities in E2F1 gene expression and/or E2F1 gene amplification have been described in various cancer cell lines and tumor types, including lung cancer [32], [33]. Of note, the overexpression of E2F1 is frequently associated with high-grade tumors and poor patient survival prognosis [29], [31], [34], suggesting that its oncogenic properties extend beyond the ability to stimulate the aberrant growth of neoplastic cells. Consistent with these findings, the latest evidence has uncovered that E2F1 is most relevant for cancer metastasis and chemoresistance [18], [19], [35]. Here, we show that the expression of E2F1 is high in lung cancer. Meanwhile, we determined that miR-493 directly targets and inhibits E2F1protein expression. A dual-luciferase reporter analysis indicated that miR-493 could bind to the sequence at the 3′-UTR of E2F1 (figure 4B). In addition, the introduction of miR-493 diminished the expression of cellular E2F1 mRNA and protein (figure 5C, D).Whereas, when inhibiting oligonucleotides against miR-493 was were transfected into HBE, A549 and H1277 cells, an inverse expression pattern was observed between miR-493 and E2F1 protein (figure 6 B). Because E2F1 plays a significant role in the regulation of cell proliferation, survival and invasion, we investigated whether E2F1 contributes to the effect of miR-493 on these phenotypes of lung cancer cells. We constructed siRNA fragments targeting E2F1 to knock down the expression of E2F1, and found that the knock-down of E2F1 could partly simulate the cell growth (figure 5 A) and cell invasion (figure 5 D, E) phenotype induced by the overexpression of miR-493. Furthermore, the overexpression of E2F1 (without an endogenous 3′-UTR) rescued the inhibition of cell growth and invasion caused by miR-493 (figure 5B,D and E).

RETRACTED

A recent study indicated that E2F1-dependent tumor progression was mediated by the activation of the cytoplasmic Ras/Raf signaling cascades [19], such as the MEK-ERK and PI3K/AKT pathway, most of which regulate cell proliferation, survival and invasion. In this study, we showed that miR-493 can inhibit the constitutive activity of AKT and ERK pathways by targeting E2F1. Subsequently, rescue experiments indicated that the miR-493-induced downregulation of E2F1 was rescued upon the introduction of E2F1 (figure 3B), and the phosphorylation levels of AKT and ERK were altered in a similar manner. These observations suggest that miR-493 inhibits the AKT and ERK pathways by targeting E2F1.

Taken together, the data from our study suggested that miR-493 may be a potential tumor suppressive miRNA that inhibits cell invasion and proliferation by blocking E2F1 in lung cancer, and subsequently suppresses the downstream AKT and ERK signaling pathways, to control cell proliferation, invasion and tumorigenesis. However, future studies will have to detect more candidate targets in additional cancer types to completely clarify the function of miR-493 in tumorigenesis.

## Materials and Methods

### Cell lines and culture

Human lung cancer cell lines (H1975, A549, H1299, H446), MRC5, a normal diploid human cell line of lung fibroblasts, and immortalized human bronchial epithelial cells HBE were obtained from and maintained as recommended by the American Type Culture Collection (ATCC, Manassas,VA, USA).The human lung cancer cell line 95D was obtained from the Cell Bank of the Chinese Academy of Sciences (Shanghai, China). The H1975, A549, H1299, H446, HBE and 95D cells were maintained in RPMI-1640 medium (Hyclone, USA), supplemented with 10% fetal bovine serum (FBS; Hyclone, USA). The MRC5 cells were maintained in DMEM medium (Hyclone, USA), supplemented with 10% fetal bovine serum (FBS; Hyclone, USA).The cells were incubated in an atmosphere of 5% CO2 at 37°C.

### Patient samples

All tissue specimens were collected via surgical resection from patients diagnosed between March 2009 and March 2012 at the Affiliated Tumor Hospital of Guangzhou Medical University (Guangzhou, Guangdong, China). Written informed consent was obtained from all study participants. The study protocol was approved by the Ethics Committee of GuangZhou Medical University.

### Reverse transcriptase (RT)-PCR and qRT-PCR

The total RNA was extracted from cells or tissues using Trizol reagent (Invitrogen, Carlsbad, CA, USA), and the RT reactions were performed using a miR-493 specific primer. The specific stem–loop RT primers for miR-493 and U6 were purchased from Ribobio co., Ltd (Guangzhou, China). The primer sequences of E2F1 were defined as follows: Forward primer: 5′-CCCATCCCAGGAGGTCACTT-3′; Reverse primer: 5-CTGCAGGCTCACTGCTCTC-3′. The primer sequences of GAPDH were defined as follows: Forward primer: 5′-CCACATCGCTCAGACACCAT-3′; Reverse primer: 5′-TGACAAGCTTCCCGTTCTCA-3′. Real-time PCR was performed using a standard protocol for the SYBR Green PCR kit (Toyobo, Osaka, Japan). U6 and GAPDH were used as references for the miRNAs and mRNAs, respectively. The 2^−ΔΔCt^ method was used to determine the relative quantities of gene expression. Each sample was analyzed in triplicate.

RETRACTED

### Western blot analysis

The protein concentration in the lysates was measured with the Protein BCA Assay Kit (Bio-Rad), and 30 ug of protein mixed with 2× SDS loading buffer was loaded per lane. The proteins in the lysates were separated by 10% SDS-PAGE and transferred to polyvinylidene difluoride membranes (Millipore). Next, the membranes were incubated for 12 hours at 4°C with an antiserum containing antibodies against E2F1, p-ERK, andβ-actin purchased from Cell signaling Technology, Akt, p-Akt, GSK3β and p-GSK3β and ERK purchased from Sigma-Aldrich Technology. A peroxidase-conjugated secondary antibody and ECL western blotting detection reagents were used to visualisethe target proteins (ECL New England Biolabs), which were quantified with a Bio Image Intelligent Quantifier 1-D (Version 2.2.1, Nihon-BioImage Ltd.). An anti-β-actin antibody was used as a protein loading control.

### Immunohistochemistry

The tissue slides included 65 primary lung samples and corresponding normal lung epithelial tissues. Immunohistochemistry was performed on formalin-fixed paraffin-embedded tissue using anti-E2F1 antibody (Cell signaling Technology) and the standard streptavidin–peroxidase staining method (Biotin-Streptavidin (ABC) IHC detection kits, Abcam Inc, US). Immunohistochemistry results were scored according to the intensity (0–4) and percentage of positive cells score 0: no staining; 1: 10% positive cells; 2: 11–50% positive cells; 3: 51–75% positive cells; 4: .75% positive cells.The relative expression was obtained by multiplying the intensity by the percentage.

### Luciferase reporter assay

A pmirGLO Dual-Luciferase miRNA target expression vector was used for the 3′-UTR luciferase assays (Promega). The target genes of miRNA-493 were selected based on the target scan algorithms [microRNA.org (http://www.microrna.org/microrna/home.do) and TargetScan (http://www.targetscan.org/)]. The primer sequences used were defined as follows: E2F1 forward primer: GC**CTCGAG**GAGATGCTCACCTTGTCTCTG, the reverse primer: CTAGCGGCCGCTGGATCTGCTTTTGAGTT. Mutant E2F1 forward primer: GAGGTGAGTGGGG*ACAAGG*CTGATGTGGGCAGGAGGGGTG, Mutant E2F1 reverses primer: CCTGCCCACATCAGCCTTGTCCCCACTCACCTCTCCCATCTC. Bold indicates the XhoI (**CTCGAG**), and underline indicates the NotI internal site. Italic (wild: **GACCTTCA** , mutant: **ACAAGG** ) indicates the target sequence. For the 3′-UTR luciferase assay, 293T cells were cotransfected with hsa-miR-493 and pmirGLO Dual-Luciferase miRNA target expression vectors with wild-type or mutant target sequence using Lipofectamine 2000.The luciferase assay was conducted using the Dual-Luciferase Reporter Assay System (Promega) 48 hours after transfection. The data are presented as the mean value ± SD for triplicate experiments and compared with the level of wild-type sequence vectors obtained in mutant-type sequence vector transfected cells that are normalized to 100%.

RETRACTED

### Lentivirus production and infection

To construct a vector expressing miR-493, the precursor sequence of miR-493 (MI0003132) was synthesized, annealed and then inserted into the BamHI–HindIII fragment of the pGCI-L3 vector (GeneCopoeia, Inc., Rockville, MD USA).The lentivirus plasmids were co-transfected with pLP1, pLP2, and pLP/VSVG (GeneCopoeia, Inc., Rockville, MD USA) into 293T cells (Invitrogen), and the virus-containing supernatants were prepared according to manufacturer's instructions. For lentivirus infection, the cells were incubated with virus-containing supernatants in the presence of 6 µg/ml polybrene. The infected cells were selected in the presence of 2 µg/ml puromycin to generate two paired stable monoclonal cell lines (a stable cell line expressing miR-493, 95D-miR-493, H1975-miR-493 and their control stable cell line, 95D -control or H1975- control). Flow cytometry analyses (FacsCalibur, Becton Dickinson) were performed on cells infected with GFP-expressing viruses for miRNA expression to confirm that 90% of cells were infected.

### Cell proliferation assay

The cells were seeded in 12-well plates at the desired cell concentrations and maintained in medium containing 10% FBS. The absorption value of cells was measured at the indicated time points in triplicate and their growth rates were recorded.

For the plate colony assay, lung cancer cells were trypsinized reseeded in 6-well plates (5–10×10^2^/well), and cultured at 37°C for 2 weeks. The cells were fixed with cold methanol at −20°C for 30 min and then stained with crystal violet (0.1%). Colonies containing more than 50 cells were counted using an imaging system (Syngene) and three independent experiments were analyzed.

RETRACTED

### E2F1 silencing

The sense sequence of siRNA oligonucleotides targeting the E2F1 transcripts (including 3 different oligonucleotides fragments) were purchased from Ribobio co., Ltd (Guangzhou, China). Scrambled siRNA was used as a negative control. The siRNA sequences for targeting E2F1 gene are defined as follows: SiRNA1: 5′-CCUGAUGAAUAUCUGUACU-3′, SiRNA2: 5′-UGGACCACCUGAUGAAUAU-3′, SiRNA3: 5′-GAGAAGUCACGCUAUGAGA-3′, siRNA controls:5′-UUGAGGUCGCGAUGGAACG-3.Cells were plated in culture dishes for 24 hours and transfected with siRNA using Lipofectamine 2000. After 48 hours, the cells were harvested for use in other assays or for RNA and protein extraction.

### E2F1-expressing vector

Full-length E2F1 cDNA entirely lacking the 3′-UTR was purchased from GeneCopeia (Rockville, MD, USA) and subcloned into the eukaryotic expression vector pcDNA3.1(+) (Invitrogen). The empty pcDNA3.1 (+) vector was used as a negative control.

### Flow cytometry analysis

The cells (1×10^6^) were digested with a trypsin solution, then harvested and washed twice with cold PBS. The washed cells were re-suspended in 0.6 mL PBS, and fixed by addition of 1.4 mL 70% v/v ethanol at 4°C overnight. The fixed cells were rinsed twice with PBS, and re-suspended in a propidium iodine solution comprising containing 40 ug/mL propidium iodine and 100 lg/mL RNaseA (Sigma-Aldrich) in PBS without calcium and magnesium, then incubated at 37°C for 30 min in the dark. The stained cells were passed through a nylon mesh sieve to remove cell clumps, and then analyzed with FACScan flow cytometer and the CELL QUEST analysis software (Becton Dickinson, San Jose, CA, USA). The flow cytometry analysis was repeated three times.

### Migration assay

The cell invasion and migration were examined with a wound-healing assay. A wound was formed by scraping the cells with a 200 mL pipette tip and washed twice with medium. We observed cells 0 and 48 hours after scraping and photographed the cells with a microscope, and the photographs were taken using an inverted microscope (Olympus) after 48 hours.

The cell invasion assay was conducted as described previously [36]. Briefly, cells were seeded onto the basement membrane matrix present in the insert of a 24-well culture plate (EC matrix; Chemicon). After an additional 48 hours, the noninvading cells and EC matrix were gently removed with a cotton swab. The invasive cells located on the lower side of the chamber were stained with crystal violet, counted, and imaged.

### In vivo tumorigenesis and metastasis assays

To evaluate the role of miR-493b in tumor formation and growth, 95D cells stably overexpressing miR-493 or a scramble control were propagated and inoculated subcutaneously into the dorsal flanks of nude mice (2×10^6^ cells in 0.2 ml volume). The tumor size was measured every 3 days. After 21 days, the mice were killed by cervical dislocation after inhalation isoflurane, necropsies were performed and the tumors were weighed. The tumor volumes were determined according to the following formula: A×B^2^/2, where A is the largest diameter and B is the diameter perpendicular to A. The experiments were performed using five or six mice per group.

RETRACTED

For the metastasis assays, lung cancer cells were injected into the tail veins of five week-old mice. On day-28, all animals were sacrificed by cervical dislocation after inhalation isoflurane, and the lung were excised. The lung metastasis images were obtained with a Bruker Small Animal Imaging System (Germany). The lung tissue was removed, fixed, paraffin-embedded, serially sectioned, and subjected to hematoxylin and eosin (H&E) staining. This study was conducted with the approval of the ethical committee of Guanzhou Medical University, Guanzhou, China, and all experimental procedures were performed in accordance with the National Institutes of Health Guide for Care and Use of Laboratory Animals (Publication No. 85-23, revised 1985).

### Statistical analysis

The data are expressed as the mean ± standard error of the mean (SEM) from at least three independent experiments. The values for the capillary tube formation and luciferase activity assays were obtained from three independent experiments performed in duplicate. Unless otherwise noted, the differences between groups were analyzed using Student's t test when only two groups were compared or using a one-way ANOVA when more than two groups were compared. All statistical tests were two-sided. The differences were considered statistically significant at P<0.05. All analyses were performed using SPSS software (SPSS Inc., Chicago, IL).
